The article "A Novel Theoretical Investigation of the Abu-Shady–Kaabar Fractional Derivative as a Modeling Tool for Science and Engineering" was published in 2022. Journal: Comput Math Methods Med.

# A Novel Theoretical Investigation of the Abu-Shady–Kaabar Fractional Derivative as a Modeling Tool for Science and Engineering

**DOI:** 10.1155/2022/4119082

**Published:** 2022-09-26

**Authors:** Francisco Martínez, Mohammed K. A. Kaabar

**Affiliations:** ^1^Department of Applied Mathematics and Statistics, Technological University of Cartagena, Cartagena 30203, Spain; ^2^Gofa Camp, Near Gofa Industrial College and German Adebabay, Nifas Silk-Lafto, Addis Ababa 26649, Ethiopia; ^3^Institute of Mathematical Sciences, Faculty of Science, Universiti Malaya, Kuala Lumpur 50603, Malaysia

## Abstract

A newly proposed generalized formulation of the fractional derivative, known as Abu-Shady–Kaabar fractional derivative, is investigated for solving fractional differential equations in a simple way. Novel results on this generalized definition is proposed and verified, which complete the theory introduced so far. In particular, the chain rule, some important properties derived from the mean value theorem, and the derivation of the inverse function are established in this context. Finally, we apply the results obtained to the derivation of the implicitly defined and parametrically defined functions. Likewise, we study a version of the fixed point theorem for *α*-differentiable functions. We include some examples that illustrate these applications. The obtained results of our proposed definition can provide a suitable modeling guide to study many problems in mathematical physics, soliton theory, nonlinear science, and engineering.

## 1. Introduction

Fractional calculus is theoretically considered as a natural extension of classical differential calculus, which has attracted many researchers, both from a more theoretical point of view and for its diverse applications in sciences and engineering. Thus, from a more theoretical perspective, various definitions of fractional derivatives have been initiated. Fractional definitions try to satisfy the usual properties of the classical derivative; however, the only property inherent in these definitions is the property of linearity. On the contrary, some of the drawbacks that these derivatives present can be located in the following:

- The Riemann-Liouville derivative does not satisfy *D*_*a*_^*α*^(1) = 0, if *α* is not a natural number
- Fractional derivative statements do not possess some of the fundamental properties of classical derivatives, such as the product rule, the quotient rule, or the chain rule
- These derived proposals, in general, do not satisfy *D*^*α*^*D*^*β*^*f* = *D*^*α*+*β*^*f*
- The definition of the Caputo derivative implies that the function *f* must be differentiable in the ordinary sense

More information on this definition of fractional derivative can be found in [1, 2].

The locally formulated fractional derivative is established through certain quotients of increments. In this sense, Khalil et al. [3] introduced a locally defined derivative, called conformable derivative. Some of the inconveniences that the previous fractional derivatives presented have been successfully solved via this definition. Thus, for example, the aforementioned rules for the derivation of products and quotients of two functions or the chain rule are properties that have been satisfied by the conformable derivative. The physical and geometric meaning of the derivative is studied in [4, 5]. However, in [6], the author shows the disadvantages of using the conformable definition compared to Caputo's fractional derivative definition, to solve some fractional models.

Recently, Abu-Shady and Kaabar [7] introduced a new generalized formulation of the fractional derivative (GFFD) that allows to solve analytically in a simple way some fractional differential equations, whose results agree exactly with those obtained via the Caputo and Riemann-Liouville derivatives. Also, this new definition has advantages compared to the conformable derivative definition. In addition, the study in [7] has been recently extended to study some important special functions in the sense of GFFD which are essential for modeling phenomena [8].

The GFFD definition is very important in studying various phenomena in science and engineering due to the powerful applicability of this definition in investigating many fractional differential equations in a very simple direction of obtaining analytical solutions without the need for approximate numerical methods or complicated algorithms like other classical fractional definitions. This definition is a modified version of the conformable definition to overcome all issues and advantages associated with the conformable one.

Regarding the geometric behavior of GFFD, by following the previous research study concerning the fractional cords orthogonal trajectories in the sense of conformable definition [5], GFFD can be similarly applied to the same example to interpret its geometrical meaning in more details.

One of the limitations of GFFD is that GFFD is locally defined derivative, and some future works are needed to proposed nonlocal formulation of GFFD in order to preserve the nonlocality property of fractional calculus. However, nonlocal definitions come with many associated challenges while working on solving fractional differential equations. Therefore, the future studies will work on overcoming all these challenges.

The work is constructed as follows: The GFFD and its main properties are presented in Section 2. New results on generalized *α*-differential functions are proposed in Section 3 to complete the study carried out in [7]. Some interesting applications of the results obtained on generalized *α*-differentiable functions are presented in Section 4. In particular, illustrative examples of the derivation of implicitly defined functions, of parametrically defined functions and of the application of the fixed point theorem for generalized *α*-differentiable functions are included. Some conclusions are drawn in Section 5.

## 2. Fundamental Tools

**Definition 1 (see [7]).**

A given function *f* : [0, ∞)⟶*R*, the GFFD of order , 0 < *α* ≤ 1, of *f* at t > 0 is expressed as

(1) $$\begin{array}{c} D^{\text{GFFD}}f\left(t\right)=\underset{\varepsilon ⟶0}{\lim}\frac{f\left(t+\left(\Gamma \left(\beta \right)/\Gamma \left(\beta -\alpha +1\right)\right)\varepsilon t^{1-\alpha }\right)-f\left(t\right)}{\varepsilon },\beta >-1,\beta \in R^{+}. \end{array}$$

If f is *α*-differentiable (*α* − DF) in some (0, a), a > 0, and $\underset{t⟶0^{+}}{\lim}D^{\text{GFFD}}f\left(t\right)$ exists, then we have

(2) $$\begin{array}{c} D^{\text{GFFD}}f\left(0\right)=\underset{t⟶0^{+}}{\lim}D^{\text{GFFD}}f\left(t\right). \end{array}$$

**Theorem 1 (see [7]).**

Let 0 < *α* ≤ 1, *β* > −1, *β* ∈ *R*^+^ and let *f*, *g* be *α* − DF at a point *t* > 0. Then, we obtain

- *D*^GFFD^[*f* + *g*] = *a* *D*^GFFD^[*f*] + *b* *D*^GFFD^[*g*], ∀*a*, *b* ∈ *R*
- *D*^GFFD^[*t*^*p*^] = (*p*Γ(*β*)/Γ(*β* − *α* + 1))*t*^*p*−*α*^, ∀*p* ∈ *R*
- *D*^*GFFD*^[*ψ*] = 0, ∀constant functions *f*(*t*) = *ψ*
- *D*^GFFD^[fg] = fD^GFFD^[*g*] + gD^GFFD^[*f*]
- *D*^GFFD^[(*f*/*g*)] = (gD^GFFD^[*f*] − fD^GFFD^[*g*]/*g*^2^)
- If, additionally, *f* is a differentiable function, then *D*^GFFD^*f*(*t*) = (Γ(*β*)/Γ(*β* − *α* + 1))*t*^1−*α*^(df/dt)(*t*).

The generalized *α*-derivative of certain functions using GFFD is expressed as:

- *D*^GFFD^[1] = 0
- *D*^GFFD^[sin(kt)] = (*k*Γ(*β*)/Γ(*β* − *α* + 1))*t*^1−*α*^cos(kt)
- *D*^GFFD^[cos(kt)] = −(*k*Γ(*β*)/Γ(*β* − *α* + 1))*t*^1−*α*^sin(kt)
- *D*^GFFD^[*e*^kt^] = (*k*Γ(*β*)/Γ(*β* − *α* + 1))*t*^1−*α*^*e*^kt^

In addition, it is interesting to highlight the generalized *α*-derivative of the following functions:

- *D*^GFFD^[(Γ(*β* − *α* + 1)/*α*Γ(*β*))*t*^*α*^] = 1
- *D*^GFFD^[sin((Γ(*β* − *α* + 1)/*α*Γ(*β*))*t*^*α*^)] = cos((Γ(*β* − *α* + 1)/*α*Γ(*β*))*t*^*α*^)
- *D*^GFFD^[cos((Γ(*β* − *α* + 1)/*α*Γ(*β*))*t*^*α*^)] = −sin((Γ(*β* − *α* + 1)/*α*Γ(*β*))*t*^*α*^)
- *D*^GFFD^[*e*^((Γ(*β* − *α* + 1)/*α*Γ(*β*))*t*^*α*^)^] = *e*^((Γ(*β* − *α* + 1)/*α*Γ(*β*))*t*^*α*^)^.

**Theorem 2 (Rolle's theorem for generalized α-differentiable functions) (see [7]).**

Let *a* > 0, *α* ∈ (0, 1] and *f* : [*a*, *b*]⟶*R* be a given function satisfying

- *f* is continuous on [*a*, *b*]
- *f* is generalized *α* − DF on (*a*, *b*)
- *f*(*a*) = *f*(*b*)

Then, ∃*c* ∈ (*a*, *b*), such that *D*^GFFD^*f*(*c*) = 0.

**Theorem 3 (Mean value theorem for generalized *α*-differentiable functions) (see [7]).**

Let *a* > 0, *α* ∈ (0, 1] and f : [*a*, *b*]⟶*R* be a given function satisfying

- *f* is continuous on [*a*, *b*]
- *f* is generalized *α* − DF on (*a*, *b*)

Then, ∃*c* ∈ (*a*, *b*), ∋

(3) $$\begin{array}{c} D^{\text{GFFD}}f\left(c\right)=\frac{f\left(b\right)-f\left(a\right)}{h\left(b^{\alpha }-a^{\alpha }\right)}, \end{array}$$

where *h* = (Γ(*β* − *α* + 1)/*α*Γ(*β*)).

## 3. New Results on Generalized *α-*Differentiable Functions

In this section, we establish important results that complete the theory of generalized *α*-differentiable functions, introduced in [7].

**Theorem 4 .**

If a given function f : [0, ∞)⟶*Risα* − DF at *t*_0_ > 0, 0 < *α* ≤ 1, *β* > −1, *β* ∈ *R*^+^, then *f* is continuous at *t*_0_.

**Proof**

Since

(4) $$\begin{array}{c} f\left(t_{0}+\left(\Gamma \left(\beta \right)/\Gamma \left(\beta -\alpha +1\right)\right)\varepsilon t_{0}^{1-\alpha }\right)=\frac{f\left(t_{0}+\left(\Gamma \left(\beta \right)/\Gamma \left(\beta -\alpha +1\right)\right)\varepsilon t_{0}^{1-\alpha }\right)-f\left(t_{0}\right)}{\varepsilon }\varepsilon +f\left(t_{0}\right), \end{array}$$

Then,

(5) $$\begin{array}{c} \underset{\varepsilon ⟶0}{\lim}\;f\left(t_{0}+\left(\Gamma \left(\beta \right)/\Gamma \left(\beta -\alpha +1\right)\right)\varepsilon t_{0}^{1-\alpha }\right)=\underset{\varepsilon ⟶0}{\lim}\left[\frac{f\left(t_{0}+\left(\Gamma \left(\beta \right)/\Gamma \left(\beta -\alpha +1\right)\right)\varepsilon t_{0}^{1-\alpha }\right)-f\left(t_{0}\right)}{\varepsilon }\varepsilon \right]+f\left(t_{0}\right)=f\left(t_{0}\right). \end{array}$$

Hence, *f* is continuous at *t*_0_

**Theorem 5 (Chain rule).**

Let 0 < *α* ≤ 1,  *β* > −1, *β* ∈ *R*^+^, *g* generalized *α* − *DF* at *t* > 0 and *f* differentiable at *g*(*t*) then

(6) $$\begin{array}{c} D^{\text{GFFD}}\left[f\circ g\right]\left(t\right)=f^{\prime }\left(g\left(t\right)\right)D^{\text{GFFD}}g\left(t\right). \end{array}$$

**Proof**

We prove the result following a standard limit approach. First, if the function *g* is constant in a neighborhood of *a* > 0 then *D*^GFFD^[*f*∘*g*](*t*) = 0. If *g* not is constant in a neighborhood of *a* > 0, we can find a *t*_0_ > 0 such that *g*(*t*_1_) ≠ *g*(*t*_2_) for any *t*_1_, *t*_2_ ∈ (*a* − *t*_0_, *a* + *t*_0_). Now, since *g* is continuous at *a*, for *ε* sufficiently small, we have

(7) $$\begin{array}{c} D^{\text{GFFD}}\left[f\circ g\right]\left(a\right)=\underset{\varepsilon ⟶0}{\lim}\frac{f\left(g\left(a+\left(\Gamma \left(\beta \right)/\Gamma \left(\beta -\alpha +1\right)\right)\varepsilon a^{1-\alpha }\right)\right)-f\left(g\left(a\right)\right)}{\varepsilon }=\underset{\epsilon ⟶0}{\lim}\frac{f\left(g\left(a+\left(\Gamma \left(\beta \right)/\Gamma \left(\beta -\alpha +1\right)\right)\varepsilon a^{1-\alpha }\right)\right)-f\left(g\left(a\right)\right)}{g\left(a+\left(\Gamma \left(\beta \right)/\Gamma \left(\beta -\alpha +1\right)\right)\varepsilon a^{1-\alpha }\right)-g\left(a\right)}∙\frac{g\left(a+\left(\Gamma \left(\beta \right)/\Gamma \left(\beta -\alpha +1\right)\right)\varepsilon a^{1-\alpha }\right)-g\left(a\right)}{\varepsilon }=\underset{\epsilon ⟶0}{\lim}\frac{f\left(g\left(a+\left(\Gamma \left(\beta \right)/\Gamma \left(\beta -\alpha +1\right)\right)\varepsilon a^{1-\alpha }\right)\right)-f\left(g\left(a\right)\right)}{g\left(a+\left(\Gamma \left(\beta \right)/\Gamma \left(\beta -\alpha +1\right)\right)\varepsilon a^{1-\alpha }\right)-g\left(a\right)}\underset{\epsilon ⟶0}{∙\lim}\frac{g\left(a+\left(\Gamma \left(\beta \right)/\Gamma \left(\beta -\alpha +1\right)\right)\varepsilon a^{1-\alpha }\right)-g\left(a\right)}{\varepsilon }. \end{array}$$

Making

(8) $$\begin{array}{c} h=g\left(a+\left(\frac{\Gamma \left(\beta \right)}{\Gamma \left(\beta -\alpha +1\right)}\right)\varepsilon a^{1-\alpha }\right)-g\left(a\right), \end{array}$$

in the first factor, so we have

(9) $$\begin{array}{c} \underset{\epsilon ⟶0}{\lim}\frac{f\left(g\left(a+\left(\Gamma \left(\beta \right)/\Gamma \left(\beta -\alpha +1\right)\right)\varepsilon a^{1-\alpha }\right)\right)-f\left(g\left(a\right)\right)}{g\left(a+\left(\Gamma \left(\beta \right)/\Gamma \left(\beta -\alpha +1\right)\right)\varepsilon a^{1-\alpha }\right)-g\left(a\right)}=\underset{\text{h}⟶0}{\lim}\frac{f\left(g\left(a\right)+h\right)-f\left(g\left(a\right)\right)}{h}, \end{array}$$

from here

(10) $$\begin{array}{c} D^{\text{GFFD}}\left[f\circ g\right]\left(a\right)=\underset{h⟶0}{\lim}\frac{f\left(g\left(a\right)+\varepsilon \right)-f\left(g\left(a\right)\right)}{h}\underset{\epsilon ⟶0}{\lim}\frac{g\left(a+\left(\Gamma \left(\beta \right)/\Gamma \left(\beta -\alpha +1\right)\right)\varepsilon a^{1-\alpha }\right)-g\left(a\right)}{\varepsilon }=f^{\prime }\left(g\left(a\right)\right)D^{\text{GFFD}}g\left(a\right). \end{array}$$

**Remark 1 .**

Using the fact that differentiability implies generalized *α*-differentiability and assuming *g*(*t*) > 0, Equation (6) can be written as

(11) $$\begin{array}{c} D^{\text{GFFD}}\left[f\circ g\right]\left(t\right)=\frac{\Gamma \left(\beta -\alpha +1\right)}{\Gamma \left(\beta \right)}g{\left(t\right)}^{\alpha -1}D^{\text{GFFD}}f\left(g\left(t\right)\right)D^{\text{GFFD}}g\left(t\right). \end{array}$$

**Theorem 6 (Extended mean value theorem for generalized *α*-differentiable functions) [5].**

Let *a* > 0, *α* ∈ (0, 1], and *f*, *g* : [*a*, *b*]⟶*R* be functions satisfying

- *f*, *g* are continuous on [*a*, *b*]
- *f*, *g* are generalized *α* − DF on (*a*, *b*)
- *D*^GFFD^*g*(*t*) ≠ 0∀*t* ∈ (*a*, *b*)
- *g*(*b*) ≠ *g*(*a*)
- *D*^GFFD^*f*(*t*) and *D*^GFFD^*g*(*t*) not annulled simultaneously on (*a*, *b*)

Then, ∃*c* ∈ (*a*, *b*), ∋

(12) $$\begin{array}{c} \frac{D^{\text{GFFD}}f\left(c\right)}{D^{\text{GFFD}}g\left(c\right)}=\frac{f\left(b\right)-f\left(a\right)}{g\left(b\right)-g\left(a\right)}. \end{array}$$

**Proof**

Consider the function

(13) $$\begin{array}{c} F\left(t\right)=f\left(t\right)-f\left(a\right)-\left(\frac{f\left(b\right)-f\left(a\right)}{g\left(b\right)-g\left(a\right)}\right)\left(g\left(t\right)-g\left(a\right)\right). \end{array}$$

Since *F* is continuous on [*a*, *b*], generalized *α* − *DF* on (*a*, *b*), and *F*(*a*) = *F*(*b*) = 0, then by Theorem 3, ∃*c* ∈ (*a*, *b*) such that *D*^*GFFD*^*F*(*c*) = 0. Using the linearity of *D*^GFFD^ and the fact that the generalized *α*-derivative of a constant is zero, our result follows.

**Remark 2 .**

Observe that Theorem 4 is a special case of this theorem for *g*(*t*) = (Γ(*β* − *α* + 1)/*α*Γ(*β*))*t*^*α*^

**Theorem 7 .**

Let *a* > 0, *α* ∈ (0, 1] and *f* : [*a*, *b*]⟶*R* be a given function satisfying

- *f* is continuous on [*a*, *b*]
- *f* is generalized *α* − DF on (*a*, *b*)

If *D*^GFFD^*f*(*t*) = 0, for all *t* ∈ (*a*, *b*), then, *f* is a constant on [*a*, *b*]

**Proof**

Suppose *D*^GFFD^*f*(*t*) = 0 for all *t* ∈ (*a*, *b*). Let *t*_1_, *t*_2_ ∈ [*a*, *b*] with *t*_1_ < *t*_2_. So, the closed interval [*t*_1_, *t*_2_] is contained in [*a*, *b*], and the open interval (*t*_1_, *t*_2_) is contained in (*a*, *b*).

Hence, *f* is continuous on [*t*_1_, *t*_2_] and *α* − DF on (*t*_1_, *t*_2_). So, by Theorem 4, there is *c* ∈ (*t*_1_, *t*_2_) with

(14) $$\begin{array}{c} \frac{f\left(t_{2}\right)-f\left(t_{1}\right)}{\left(\Gamma \left(\beta -\alpha +1\right)/\alpha \Gamma \left(\beta \right)\right)\left(t_{2}^{\alpha }-t_{1}^{\alpha }\right)}=D^{\text{GFFD}}f\left(c\right)=0. \end{array}$$

Therefore, *f*(*t*_2_) − *f*(*t*_1_) = 0 and *f*(*t*_2_) = *f*(*t*_1_)

Since *t*_1_ and *t*_2_ are arbitrary numbers in [*a*, *b*] with *t*_1_ < *t*_2_, then *f* is a constant on [*a*, *b*].

**Corollary 1 (see [5]).**

Let *a* > 0, *α* ∈ (0, 1], and *F*, *G* : [*a*, *b*]⟶*R* be functions such that *D*^GFFD^*F*(*t*) = *D*^GFFD^*G*(*t*)∀*t* ∈ (*a*, *b*). Then, ∃ a constant C such that

(15) $$\begin{array}{c} F\left(t\right)=G\left(t\right)+C. \end{array}$$

**Proof**

By simply applying the above theorem to *H*(*t*) = *F*(*t*) − *G*(*t*), it can easily be proven.

**Theorem 8 (see [5]).**

Let a > 0, *α* ∈ (0, 1], and f : [*a*, *b*]⟶*R* be a given function satisfying

- *f* is continuous on [*a*, *b*]
- f is generalized *α* − DF on (*a*, *b*)

Then, we have

- If *D*^GFFD^*f*(*t*) > 0∀t ∈ (*a*, *b*), then *f* is strictly increasing on [*a*, *b*]
- If *D*^GFFD^*f*(*t*) < 0∀t ∈ (*a*, *b*), then *f* is strictly decreasing on [*a*, *b*]

**Proof**

Following similar line of argument as given in the Theorem 10, there exists *c* between *t*_1_ and *t*_2_ with

(16) $$\begin{array}{c} \frac{f\left(t_{2}\right)-f\left(t_{1}\right)}{\left(\Gamma \left(\beta -\alpha +1\right)/\alpha \Gamma \left(\beta \right)\right)\left(t_{2}^{\alpha }-t_{1}^{\alpha }\right)}=D^{\text{GFFD}}f\left(c\right). \end{array}$$

1. If *D*^GFFD^*f*(*c*) > 0, then *f*(*t*_2_) > *f*(*t*_1_) for *t*_1_ < *t*_2_. Therefore, *f* is strictly increasing on [*a*, *b*], since *t*_1_ and *t*_2_ are arbitrary number of [*a*, *b*]
2. If *D*^GFFD^*f*(*c*) < 0, then *f*(*t*_2_) < *f*(*t*_1_) for *t*_1_ < *t*_2_. Therefore, *f* is strictly decreasing on [*a*, *b*], since *t*_1_ and *t*_2_ are arbitrary number of [*a*, *b*].

**Definition 2 .**

Let I ⊂ (0, ∞) an open interval, *α* ∈ (0, 1], and *f* : *I*⟶*R* be we will say that *f* ∈ *C*^*α*^(*I*, *R*) if the f is generalized *α* − DF  on *I* and generalized *α*-derivative is continuous on *I*.

**Theorem 9 .**

Let *I* ⊂ (0, ∞) an open interval, *α* ∈ (0, 1], and *f* : *I*⟶*R* be a function of class *C*^*α*^ on the interval I. Suppose *f*(*a*) = *b* for some *a* ∈ I, and *D*^GFFD^*f*(*a*) ≠ 0. Then, there is an open neighborhood *U* of *a* in which *f* admits an inverse function *f*^−1^ of class *C*^*α*^ on the open neighborhood *V* = *f*(*U*) of *b*, and its generalized *α*-derivative is

(17) $$\begin{array}{c} D^{\text{GFFD}}f^{-1}\left(y\right)={\left(\frac{\Gamma \left(\beta \right)}{\Gamma \left(\beta -\alpha +1\right)}\right)}^{2}\frac{t^{1-\alpha }y^{1-\alpha }}{D^{GFFD}f\left(t\right)},\forall y\in V,t=f^{-1}\left(y\right). \end{array}$$

**Proof**

Since *D*^GFFD^*f*(*t*) is continuous in the open interval *I*, it is a known fact that there exists an open neighborhood *U* of *a* in which *D*^GFFD^*f*(*t*) has a constant sign (the sign of *D*^GFD^*f*(*a*)). From Theorem 14, it follows *f* that is strictly monotonic on *U* (increasing if *D*^GFFD^*f*(*a*) > 0 and decreasing if *D*^GFFD^*f*(*a*) < 0). Therefore, *f* is continuous and strictly monotonic on *U*, so there is the inverse function of the one-to-one function *f* : *U*⟶*V*, with *V* = *f*(*U*). This inverse *f*^−1^ : *V*⟶*U* is of class *C*^*α*^ and strictly monotonic (in the same sense that *f* is) on *V*. Equation (30) can be obtained from the identity *f*(*f*^−1^(*y*)) = *y* for all *y* ∈ *V*, in which the *α*-derivative (with respect to *y*) is calculated, applying the chain rule

(18) $$\begin{array}{c} \frac{\Gamma \left(\beta -\alpha +1\right)}{\Gamma \left(\beta \right)}t^{\alpha -1}D^{\text{GFFD}}f\left(t\right)∙D^{\text{GFFD}}f^{-1}\left(y\right)=\frac{\Gamma \left(\beta \right)}{\Gamma \left(\beta -\alpha +1\right)}y^{1-\alpha },\forall y\in V,t=f^{-1}\left(y\right). \end{array}$$

## 4. Applications

Some interesting applications of the results obtained on generalized *α* − DF functions are presented in this section.

### 4.1. Generalized **α**-Derivative of an Implicit Function

It is a known fact that an equation *F*(*t*, *y*) = 0 implicitly defines a function *y* = *g*(*t*) in a certain open interval *I*, if *F*(*t*, *g*(*t*)) = 0∀*t* ∈ *I*. Suppose that *g*(*t*) and *F*(*t*, *g*(*t*)) are generalized *α* − *DF* functions in an open interval *I* ⊂ (*o*.∞), then the derivative *D*^GFFD^*g*(*t*) can be found by calculating the generalized *α*-derivative of *F*(*t*, *g*(*t*)), as a compound function, and canceling this derivative calculated.

Now, we are going to calculate the derivative of the generalized 1/3-differentiable *y* = *g*(*t*) function at the point *t* = 8, such that *g*(8) = 1, and it is implicitly defined by the equation

(19) $$\begin{array}{c} \left(\sqrt[{3}]{t}-2\right)e^{6\sqrt[{3}]{y}}-3\sqrt[{3}]{\text{t}}\sin\left(1-\sqrt[{3}]{y}\right)-\sqrt[{3}]{y}+1=0. \end{array}$$

Calculating the 1/3 -derivative in this equation, we obtain

(20) $$\begin{array}{c} \frac{1}{3}\frac{\Gamma \left(\beta \right)}{\Gamma \left(\beta +2/3\right)}e^{6\sqrt[{3}]{g\left(t\right)}}+2\left(\sqrt[{3}]{t}-2\right)e^{6\sqrt[{3}]{g\left(t\right)}}g{\left(t\right)}^{-2/3}D^{\text{GFFD}}g\left(t\right)-\frac{\Gamma \left(\beta \right)}{\Gamma \left(\beta +2/3\right)}\sin\left(1-\sqrt[{3}]{g\left(t\right)}\right)+\sqrt[{3}]{\text{t}}\cos\left(1-\sqrt[{3}]{g\left(t\right)}\right)g{\left(t\right)}^{-2/3}D^{\text{GFFD}}g\left(t\right)-\frac{1}{3}g{\left(t\right)}^{-2/3}D^{\text{GFFD}}g\left(t\right)=0. \end{array}$$

Taking *t* = 8 and *g*(8) = 1 in the equation above, we have

(21) $$\begin{array}{c} \frac{1}{3}\frac{\Gamma \left(\beta \right)}{\Gamma \left(\beta +2/3\right)}e^{6}+2D^{\text{GFFD}}g\left(8\right)-\frac{1}{3}D^{\text{GFFD}}g\left(8\right)=0. \end{array}$$

Finally, the generalized 1/3-derivative is given by

(22) $$\begin{array}{c} D^{\text{GFFD}}g\left(8\right)=-\frac{\Gamma \left(\beta \right)}{\Gamma \left(\beta +2/3\right)}\frac{e^{6}}{5}. \end{array}$$

### 4.2. Generalized *α*-Derivative of a Parametrically Defined Function

Let *t* = *t*(*λ*), *y* = *y*(*λ*) be generalized *α* − *DF* functions on an open interval *I* ⊂ (*o*.∞), with *D*^GFFD^*t*(*λ*) ≠ 0∀*λ* ∈ *I*. If *t* = *t*(*λ*) and *y* = *y*(*λ*), define the function *y* = *y*(*λ*(*t*)) = *y*(*t*) (where *λ*(*t*) is the inverse function of *t*(*λ*)), and then, the generalized *α*-derivative of this function is given by

(23) $$\begin{array}{c} D^{\text{GFFD}}y\left(t\right)=\frac{\Gamma \left(\beta -\alpha +1\right)}{\Gamma \left(\beta \right)}∙\lambda^{\alpha -1}∙D^{\text{GFFD}}y\left(\lambda \right)∙D^{\text{GFFD}}\lambda \left(t\right)=\frac{\Gamma \left(\beta -\alpha +1\right)}{\Gamma \left(\beta \right)}∙\lambda^{\alpha -1}∙D^{\text{GFFD}}y\left(\lambda \right)∙{\left(\frac{\Gamma \left(\beta \right)}{\Gamma \left(\beta -\alpha +1\right)}\right)}^{2}∙\frac{\lambda^{1-\alpha }t^{1-\alpha }}{D^{\text{GFFD}}t\left(\lambda \right)}=\frac{\Gamma \left(\beta \right)}{\Gamma \left(\beta -\alpha +1\right)}\frac{D^{\text{GFFD}}y\left(\lambda \right)}{D^{\text{GFFD}}t\left(\lambda \right)}{\left(t\left(\lambda \right)\right)}^{1-\alpha }. \end{array}$$

Note that the above expression is obtained by applying the chain rule and the derivation formula of the inverse function, both in the generalized sense.

Thus, for example, consider the function *y* = *y*(*t*) defined parametrically by

(24) $$\begin{array}{c} \begin{array}{c} t\left(\lambda \right)=r\left(3\sqrt[{3}]{\lambda }++\sin\left(3\sqrt[{3}]{\lambda }\right)\right)\\ y\left(\lambda \right)=r\left(1-\cos\left(3\sqrt[{3}]{\lambda }\right)\right) \end{array},\forall \lambda \in \left[0,{\left(\frac{2\pi }{3}\right)}^{3.}\right], \end{array}$$

is generalized 1/3-differentiable and its 1/3-derivative is (as a function of *t*)

(25) $$\begin{array}{c} D^{\text{GFFD}}y\left(t\right)=\frac{\Gamma \left(\beta \right)}{\Gamma \left(\beta +2/3\right)}\frac{D^{\text{GFFD}}y\left(\lambda \right)}{D^{\text{GFFD}}t\left(\lambda \right)}{\left(t\left(\lambda \right)\right)}^{2/3}=\frac{\Gamma \left(\beta \right)}{\Gamma \left(\beta +2/3\right)}\frac{\sin\left(3\sqrt[{3}]{\lambda }\right)}{1+\cos\left(3\sqrt[{3}]{\lambda }\right)}\sqrt[{3}]{r^{2}{\left(3\sqrt[{3}]{\lambda }++\sin\left(3\sqrt[{3}]{\lambda }\right)\right)}^{2}}=\frac{\Gamma \left(\beta \right)}{\Gamma \left(\beta +2/3\right)}\tan\left(\frac{3\sqrt[{3}]{\lambda }}{2}\right)\sqrt[{3}]{r^{2}{\left(3\sqrt[{3}]{\lambda }++\sin\left(3\sqrt[{3}]{\lambda }\right)\right)}^{2}}. \end{array}$$

### 4.3. Fixed Point Theorem for Generalized  *α*-Derivative

We present the fixed point theorem for generalized *α*-derivative and its respective proof. In addition, we will establish some important results about the iteration of the fixed point in the generalized *α*-derivative sense. However, we first present some basic concepts and necessary results for the developments that we are going to carry out.

**Definition 3 .**

Let the following fixed-point equation *t* = *f*(*t*). Here, *f* is a mapping from *X*⟶*X*. We assume that *X* is endowed with the metric *d*. A point *t* ∈ *X* which satisfies *t* = *f*(*t*) is called a fixed point of *f*.

**Theorem 10 (Modified mean value theorem for generalized α-differentiable functions).**

Let *a* > 0, *α* ∈ (0, 1] and *f* : [*a*, *b*]⟶*R* be a given function satisfying

- *f* is continuous on [*a*, *b*]
- *f* is generalized *α* − DF on (*a*, *b*)

Then, ∃*c* ∈ (*a*, *b*), ∋

(26) $$\begin{array}{c} \frac{D^{\text{GFFD}}f\left(c\right)}{{\text{hc}}^{1-\alpha }}=\frac{f\left(b\right)-f\left(a\right)}{b-a}, \end{array}$$

where *h* = (Γ(*β*)/Γ(*β* − *α* + 1)).

**Proof**

Consider the function

(27) $$\begin{array}{c} g\left(t\right)=f\left(t\right)-f\left(a\right)-\frac{f\left(b\right)-f\left(a\right)}{b-a}\left(t-a\right). \end{array}$$

Then, the function *g* satisfies the conditions of Theorem 3. Hence, ∃*c* ∈ (*a*, *b*), ∋_0_^*C*^*T*_*t*_^*α*^[*g*](*c*) = 0. Therefore

(28) $$\begin{array}{c} 0=D^{\text{GFFD}}g\left(c\right)=D^{\text{GFFD}}f\left(c\right)-\frac{f\left(b\right)-f\left(a\right)}{b-a}∙\frac{\Gamma \left(\beta \right)}{\Gamma \left(\beta -\alpha +1\right)}∙c^{1-\alpha }. \end{array}$$

Hence,

(29) $$\begin{array}{c} \frac{{\text{D}}^{\text{GFFD}}f\left(c\right)}{{\text{hc}}^{1-\alpha }}=\frac{f\left(b\right)-f\left(a\right)}{b-a}. \end{array}$$

Now, we establish the fixed point theorem for generalized  *α*-derivative.

**Theorem 11 .**

Let *a* > 0 and *α* ∈ (0, 1]. If *f* ∈ *C*([*a*, *b*], *R*)  and *f*(*t*) ∈ [*a*, *b*], ∀*t* ∈ [*a*, *b*], then *g* has a fixed point at [*a*, *b*]. If also, *f* is generalized *α* − *DF* on (*a*, *b*) and

(30) $$\begin{array}{c} \left|\frac{\Gamma \left(\beta -\alpha +1\right)}{\Gamma \left(\beta \right)}\frac{D^{GFFD}f\left(t\right)}{t^{1-\alpha }}\right|\leq k<1,\forall t\in \left(a,b\right), \end{array}$$

then *f* has a unique fixed point p at [*a*, *b*].

**Proof**

If *f*(*a*) = *a* or *f*(*b*) = *b*, the existence of the fixed point is obvious. Suppose that *f*(*a*) ≠ *a* and *f*(*b*) ≠ *b*, therefore *f*(*a*) > *a* and *f*(*b*) < *b*. Let *g*(*t*) = *f*(*t*) − *t*, clearly continuous on [*a*, *b*], we have

(31) $$\begin{array}{c} g\left(a\right)=f\left(a\right)-a>0\text{ and }g\left(b\right)=f\left(b\right)-b<0. \end{array}$$

By the classical intermediate value theorem, then ∃*p* ∈ (*a*, *b*)∋*g*(*p*) = 0; that is

(32) $$\begin{array}{c} g\left(p\right)=f\left(p\right)-p=0. \end{array}$$

Therefore, *f* has a fixed point at *p*.

Suppose also that Equation (30) is satisfied and that *p* and *q* are fixed points on [*a*, *b*] with *p* ≠ *q*. By Theorem 16, ∃ is a number *ξ* between *p* and *q*, and therefore, in (*a*, *b*), such that

(33) $$\begin{array}{c} \left|p-q\right|=\left|f\left(p\right)-f\left(q\right)\right|=\left|\frac{\Gamma \left(\beta -\alpha +1\right)}{\Gamma \left(\beta \right)}\frac{D^{\text{GFD}}f\left(\xi \right)}{\xi^{1-\alpha }}\right|\left|p-q\right|\leq k\left|p-q\right|<\left|p-q\right|, \end{array}$$

which implies that |*p* − *q*| < |*p* − *q*| which is contradiction, therefore *p* = *q*.

**Remark 3 .**

To approximate the fixed point of a function *f*, we choose an initial approximate value *p*_0_, and we obtain the succession {*p*_*n*_}_*n*=0_^∞^ by taking *p*_*n*_ = *f*(*p*_*n*−1_) for each *n* ≥ 1. If the succession {*p*_*n*_}_*n*=0_^∞^ of converges *p* and *f* is a continuous function, then

(34) $$\begin{array}{c} p=\underset{n⟶\infty }{\lim}p_{n}=\underset{n⟶\infty }{\lim}f\left(p_{n-1}\right)=f\left(\underset{n⟶\infty }{\lim}p_{n-1}\right)=f\left(p\right), \end{array}$$

and a solution of the equation *t* = *f*(*t*) is obtained. This technique is called iterative technique of the fixed point or functional iteration.

The following result provides a first step to determine a procedure that guarantees that the function *f* converges a solution of the equation *t* = *f*(*t*) and that also chooses *f* correctly in such a way that it makes the convergence as quickly as possible.

**Theorem 12 .**

Let *a* > 0 and *α* ∈ (0.1]. If *f* ∈ *C*([*a*, *b*], *R*) and *f*(*t*) ∈ [*a*, *b*], for all *t* ∈ [*a*, *b*]. Also, suppose that *f* is generalized *α* − *DF* on (*a*, *b*) with

(35) $$\begin{array}{c} \left|\frac{\Gamma \left(\beta -\alpha +1\right)}{\Gamma \left(\beta \right)}\frac{D^{\text{GFFD}}f\left(t\right)}{t^{1-\alpha }}\right|\leq k<1,\forall t\in \left(a,b\right). \end{array}$$

If *p*_0_ is any number in [*a*, *b*], then, the succession defined by

(36) $$\begin{array}{c} p_{n}=f\left(p_{n-1}\right),n\geq 1, \end{array}$$

converges the unique fixed point *p* in [*a*, *b*].

**Proof**

First, by Theorem 17, ∃is a unique fixed point at [*a*, *b*]. On the other hand, since *f* applies to [*a*, *b*] itself, the sequence {*p*_*n*_}_*n*=0_^∞^ is defined ∀*n* ≥ 0 and *p*_*n*_ ∈ [*a*, *b*]∀*n*. Using Equation (35) and the intermediate value theorem,

(37) $$\begin{array}{c} \left|p_{n}-p\right|=\left|f\left(p_{n-1}\right)-f\left(p\right)\right|=\left|\frac{\Gamma \left(\beta -\alpha +1\right)}{\Gamma \left(\beta \right)}\frac{D^{\text{GFFD}}f\left(\xi \right)}{\xi^{1-\alpha }}\right|\left|p_{n-1}-p\right|\leq k\left|p_{n-1}-p\right|, \end{array}$$

where *ξ* ∈ (*a*, *b*). Applying the above equation inductively results

(38) $$\begin{array}{c} \left|p_{n}-p\right|\leq k\left|p_{n-1}-p\right|\leq k^{2}\left|p_{n-2}-p\right|\leq \cdots \leq k^{n}\left|p_{0}-p\right|. \end{array}$$

Since *k* < 1, it easily follows that

(39) $$\begin{array}{c} \underset{n⟶\infty }{\lim}\left|p_{n}-p\right|\leq \underset{n⟶\infty }{\lim}k^{n}\left|p_{0}-p\right|=0, \end{array}$$

and {*p*_*n*_}_*n*=0_^∞^ converges to *p*.

**Corollary 2 .**

If *f* satisfies the hypotheses of Theorem 19, then

(40) $$\begin{array}{c} \left|p_{n}-p\right|\leq \frac{k^{n}}{1-k}\left|p_{0}-p_{1}\right|,\forall n\geq 1. \end{array}$$

**Proof**

For *n* ≥ 1, the procedure used in the proof of Theorem 19 implies that

(41) $$\begin{array}{c} \left|p_{n+1}-p_{n}\right|=\left|f\left(p_{n}\right)-f\left(p_{n-1}\right)\right|\leq k\left|p_{n}-p_{n-1}\right|\leq \cdots \leq k^{n}\left|p_{1}-p_{0}\right|. \end{array}$$

Hence, for *m* > *n* ≥ 1

(42) $$\begin{array}{c} \left|p_{m}-p_{n}\right|=\left|p_{m}-p_{m-1}+p_{m-1}-\cdots -p_{n+1}+p_{n+1}-p_{n}\right|\leq \left|p_{m}-p_{m-1}\right|+\left|p_{m-1}-p_{m-2}\right|+\cdots +\left|p_{n+1}-p_{n}\right|\leq k^{m-1}\left|p_{1}-p_{0}\right|+k^{m-2}\left|p_{1}-p_{0}\right|+k^{n}\left|p_{1}-p_{0}\right|=k^{n}\left(1+k+k^{2}+\cdots +k^{m-n-1}\right)\left|p_{1}-p_{0}\right|. \end{array}$$

By Theorem 19, $\underset{n⟶\infty }{\lim}p_{m}=p$, so

(43) $$\begin{array}{c} \left|p-p_{n}\right|=\underset{m⟶\infty }{\lim}\left|p_{m}-p_{n}\right|\leq k^{n}\left|p_{0}-p\right|\overset{\infty }{\underset{i=0}{\sum }}k^{i}=\frac{k^{n}}{1-k}\left|p_{0}-p_{1}\right|. \end{array}$$

**Remark 4 .**

It is clear that the speed of convergence depends on the factor *k*^*n*^/1 − *k*, and the smaller *k* can be made, the faster the convergence will be. Convergence can be very slow if *k* is close to 1.

Finally, we present an example that illustrates these last established results.

Consider the function: $f\left(t\right)=2^{-\sqrt{t}}$ on the interval [1/9, 1], and we take *α* = *β* = 1/2. We can observe that *f*([1/9, 1]) = [0.5,0.7937005259840997] ⊂ [1/9, 1]. Also, *f* is continuous and

(44) $$\begin{array}{c} \left|\frac{\Gamma \left(1\right)}{\Gamma \left(1/2\right)}\frac{D^{\text{GFFD}}f\left(t\right)}{\sqrt{t}}\right|=\left[-\frac{\log2}{2\sqrt{t}2^{\sqrt{t}}}\right]\leq 0.82522692269223647775,\forall t\in \left[\frac{1}{9},1\right], \end{array}$$

so *f* satisfies the hypotheses of Theorem 17 and has a unique fixed point at [1/9, 1]. In addition, if we use Corollary 20, we can estimate the number of iterations required to find an approximation of the fixed point with a precision of 10^−4^. Taking *p*_0_ = 1, to obtain this precision, 54 iterations are required. Also, note that since the generalized 1/2-derivative *D*^GFFD^*f*(*t*) is negative, the successive approximations oscillate around the fixed point.

## 5. Conclusions

Novel results regarding the Abu-Shady–Kaabar fractional derivative have been investigated in this study which are extensions of the previous research study's results in [7]. In particular, some important properties of the generalized fractional derivative have been accomplished, such as the chain rule, some consequences of the mean value theorem, and the derivation of the inverse function. It is verifiable with the fact that these newly obtained results are considered as a natural extension of the classical differential calculus. The potential of this new definition of fractional derivative, both from a theoretical point of view and due to its applications, is evident through the developments and illustrative examples included in the previous section. This research can definitely open a new path for more related future works in which the results of classical mathematical analysis are extended in the sense of this new definition of fractional derivative. This definition will be applied further in studying various partial differential equations such as Schrödinger equation and Wazwaz–Benjamin–Bona–Mahony equation to study some solutions that are important in soliton theory and many other interesting research topics. Some specific examples of studies that can be further studied in the sense of GFFD are the Klein–Fock–Gordon equation via the Kudryashov-expansion method [9], the systems of fractional-order partial differential equations via the Laplace optimized decomposition technique [10], and the noninteger fractional-order hepatitis B model [11], by comparing the previous results in the senses of conformable and Caputo definitions with new results using GFFD. Numerical experiments with error analysis including comparison between conformable derivative and our definition including CPU time in the graphical representations in the sense of our proposed definition will be conducted in our future studies. In addition, in our future study, all algorithms and/or pseudo-codes will be provided for the solutions' steps using one of the common software packages such as MAPLE and MATHEMATICA.

## Data Availability

No data were used to support this study.
